RETRACTED

# Irisin Attenuates Oxidative Stress, Mitochondrial Dysfunction, and Apoptosis in the H9C2 Cellular Model of Septic Cardiomyopathy through Augmenting Fundc1-Dependent Mitophagy

**DOI:** 10.1155/2021/2989974

**Published:** 2021-08-18

**Authors:** Xiaoqing Jiang, Shumin Cai, Yinghui Jin, Feng Wu, Jing He, Xixuan Wu, Ying Tan, Yu Wang

**Affiliations:** ^1^Department of Critical Care Medicine, Nanfang Hospital, Southern Medical University, Guangzhou 510515, China; ^2^Department of Hepatobiliary Surgery, Nanfang Hospital, Southern Medical University, Guangzhou 510515, China

## Abstract

In the present study, we used lipopolysaccharide- (LPS-) stimulated H9C2 cardiomyocytes to investigate whether irisin treatment attenuates septic cardiomyopathy via Fundc1-related mitophagy. Fundc1 levels and mitophagy were significantly reduced in LPS-stimulated H9C2 cardiomyocytes but were significantly increased by irisin treatment. Irisin significantly increased ATP production and the activities of mitochondrial complexes I and III in the LPS-stimulated cardiomyocytes. Irisin also improved glucose metabolism and significantly reduced LPS-induced levels of reactive oxygen species by increasing the activities of antioxidant enzymes, glutathione peroxidase (GPX), and superoxide dismutase (SOD), as well as levels of reduced glutathione (GSH). TUNEL assays showed that irisin significantly reduced LPS-stimulated cardiomyocyte apoptosis by suppressing the activation of caspase-3 and caspase-9. However, the beneficial effects of irisin on oxidative stress, mitochondrial metabolism, and viability of LPS-stimulated H9C2 cardiomyocytes were abolished by silencing Fundc1. These results demonstrate that irisin abrogates mitochondrial dysfunction, oxidative stress, and apoptosis through Fundc1-related mitophagy in LPS-stimulated H9C2 cardiomyocytes. This suggests irisin is a potentially useful treatment for septic cardiomyopathy, though further investigations are necessary to confirm our findings.

## 1. Introduction

Sepsis refers to excessive activation of the immune system in response to microbial infections that result in inflammation-related injury [1, 2]. Sepsis-induced myocardial injury is termed as septic cardiomyopathy, which is associated with increased morbidity and mortality. Hemodynamic imbalances in response to sepsis render the heart unable to maintain adequate preload [3]. Besides, sepsis-related cytokines promote cardiomyocyte apoptosis and endothelial cell dysfunction, both of which diminish cardiac output and vascular tone [4]. The pathogenesis of septic cardiomyopathy includes oxidative stress, calcium imbalance, mitochondrial dysfunction, endoplasmic reticulum stress, autophagy inhibition, activation of programmed cell death activation, and immune disorder [5, 6]. In our previous study, we demonstrated that cardiac dysfunction during LPS-induced sepsis involved mitochondrial fission-associated mitochondrial damage. Excessive mitochondrial fission promotes mitochondrial damage, reduced synthesis of mitochondrial ATP, and cardiomyocyte death via mitochondria-dependent apoptotic pathway, which results in reduced cardiac performance [7, 8]. Therefore, mitochondrial dysfunction is a potential molecular mechanism underlying septic cardiomyopathy [9, 10].

RETRACTED

Fundc1-dependent mitophagy is a protective mechanism that involves degradation of injured mitochondria through the lysosomes [11–14]. Mitophagy protects against cardiovascular disorders through antioxidative, antiapoptotic, and anti-inflammatory effects [15–18]. For example, hypoxia-induced mitophagy attenuates myocardial ischemia-reperfusion injury by reducing the death of cardiomyocytes [15, 19]. Mitophagy activation attenuates heart failure by increasing ATP production in the cardiomyocytes and correcting the redox balance [20]. Besides, mitophagy activation is also associated with cardiac progenitor cell differentiation and mitochondrial network remodeling [21]. Fundc1-mediated mitophagy is closely associated with inflammation through the STING pathway [22], thereby suggesting its potential role in septic cardiomyopathy.

Although protective effects of mitophagy have been widely observed, mitophagy is significantly suppressed under stressful conditions [23–25]. Therefore, several approaches have been designed to enhance mitophagy. For example, melatonin protects cardiac microvasculature against ischemia/reperfusion injury by activating mitophagy [26]. Empagliflozin is an antidiabetic drug that activates mitophagy in type-2 diabetes [27]. In our previous study, we suppressed septic cardiomyopathy by inhibiting DRP1-related mitochondrial fission using irisin [28]. In this study, we investigated if irisin treatment protects against sepsis-induced cardiomyopathy via Fundc1-related mitophagy using LPS-stimulated H9C2 cardiomyocytes as a model.

## 2. Materials and Methods

### 2.1. Cell Culture

H9C2 cardiomyocytes were purchased from the American Type Culture Collection (ATCC, Manassas, VA, USA) and cultured in DMEM medium containing 10% fetal bovine serum at 37°C and 5% CO_2_ in a humidified incubator. When the cell density reached 70%~80%, the cells were subcultured in a 1 : 3 ratio after digestion with 0.25% trypsin [29]. We induced septic cardiomyopathy *in vitro* by culturing H9C2 cells in 1 *μ*g/ml LPS for 24 h. Besides, cardiomyocyteswere treated with irisin (20 nmol/L) 24 h before LPS stress.

RETRACTED

### 2.2. MTT Assay

We incubated 1 × 10^4^/ml diluted H9C2 cells in 96-well plates at 37°C and 5% CO_2_ in a humidified incubator. The culture solution was changed every day. After incubation for 24 h, 48 h, and 72 h, respectively, the culture solution was discarded, and the cells were washed with PBS [30]. Then, 20 *μ*l of MTT solution was added to each well and incubated at 37°C for 4 h in the dark. After discarding the culture solution with MTT, we added 150 *μ*l DMSO into each well [31]. The plate was constantly shaken for 10 min to fully dissolve the purple crystals. Then, the OD values were measured in an enzyme-linked immunosorbent detector at 490 nm wavelength [32, 33].

### 2.3. Western Blotting

The transfected cells were lysed in RIPA buffer (Thermo Scientific, Belmont, MA, USA) for 30 minutes at 4°C. Equal amounts of protein samples were separated on a 10% SDS-polyacrylamide gel electrophoresis (SDS-PAGE) and transferred to PVDF membrane (Roche) by electroblotting [34, 35]. The membrane was blocked by incubation with skimmed milk at 4°C overnight. Then, the membrane was incubated with the primary antibody overnight at 4°C. GAPDH was used as internal reference and probed with anti-GAPDH antibody [36]. The membranes were incubated with HRP-conjugated secondary antibody at room temperature for 2 h. Finally, the membranes were developed using the ECL substrate reagent kit (GE Healthcare) and analyzed using the Gel Doc XR imaging system (Bio-Rad, USA). Each sample was analyzed in triplicate [37].

### 2.4. Quantitative Real-Time PCR (qRT-PCR)

Total cellular RNA was isolated using total RNA extraction reagent (R401-01, Vazyme, Nanjing) according to manufacturer's instructions [38]. Then, 1 *μ*g RNA was reversed transcribed to cDNA using Hiscript Q RT SuperMix for qPCR (R122-01, Vazyme, Nanjing) as described by manufacturer's instructions. Quantitative PCR was performed using ChamQ SYBR Master Mix (Q311-02, Vazyme, Nanjing) in a LightCycler 96 (Roche, Risch-Rotkreuz, Switzerland) with the following conditions: 5 min at 95°C, followed by 40 cycles at 95°C for 30 s, 60°C for 40 s, and 72°C for 60 s [39].

### 2.5. Immunofluorescence

The cells were fixed in formalin, dehydrated with alcohol, and blocked in PBST with 5% BSA for 1 h at RT. The cells were then incubated with primary antibodies at 4°C overnight followed by incubation with secondary antibodies for 1 h at RT [40]. Then, the samples were stained with DAPI, mounted on slides, and photographed using the Olympus microscope at 200x magnification [41, 42]. The average fluorescence intensity was calculated using Image J software. Five random fields were analyzed for every sample [43].

RETRACTED

### 2.6. Detection of Reactive Oxygen Species (ROS)

The cells were cultured in a 24-well plate. Then, after discarding the supernatant, the cells were incubated in the dark at 37°C for 20 min with 500 *μ*l medium per well containing 2,7-dichlorodihydrofluorescein diacetate (DCFH-DA, Cayman Chemical, Michigan, USA, Catalog: 85155) to detect the levels of intracellular ROS [44]. After removing the medium with the dye, cells were twice rinsed with PBS and photographed under a fluorescence microscope [45].

### 2.7. Measurement of Antioxidant Enzyme Activities

The cells were trypsinized and centrifuged at 1,000 rpm for 10 min. After removing the supernatant [46, 47], the cell pellet was resuspended in 500 *μ*l of PBS solution and homogenized by sonication for two seconds [48]. This was repeated ten times to obtain total cellular homogenate. Then, the activities of glutathione peroxidase (GSH-Px, Catalog: A005), GSH (CAT, Catalog: A007-1-1), and superoxide dismutase (SOD, Catalog: A001-3-2) were determined in the cell homogenates according to manufacturer's instructions [49].

### 2.8. Statistical Analysis

All *in vitro* experiments were performed in triplicate. All experiments were repeated three times. The experiments were performed using five rats per group. Data are presented as means ± SD and were analyzed using SPSS 23.0 software [49]. Student's *t*-test was used to compare data from two experimental groups. One-way ANOVA followed by Tukey's multiple comparisons test was used to evaluate differences between multiple groups. *p* < 0.05 was considered statistically significant.

## 3. Results

### 3.1. Irisin Activates Fundc1-Related Mitophagy in LPS-Stimulated Cardiomyocytes

We first analyzed the effects of irisin on Fundc1-related mitophagy in LPS-stimulated cardiomyocytes. Western blot analysis showed that Fundc1 protein levels were rapidly downregulated in LPS-stimulated cardiomyocytes compared to the controls (Figures 1(a) and 1(b)). However, Fundc1 protein levels were significantly higher in irisin plus LPS-stimulated cardiomyocytes compared to the LPS-stimulated cardiomyocytes alone (Figures 1(a) and 1(b)). This suggested that irisin treatment is protected against defective Fundc1-related mitophagy in LPS-stimulated cardiomyocytes. We then analyzed the status of mitophagy using immunofluorescence. LPS treatment significantly reduced mitophagy compared to the control group, but these effects were reversed by irisin (Figures 1(c) and 1(d)). Taken together, these results demonstrated that Fundc1-related mitophagy was activated by irisin in LPS-stimulated cardiomyocytes.

### 3.2. Irisin Enhances ATP Production and Mitochondrial Metabolism through Fundc1-Related Mitophagy in LPS-Stimulated Cardiomyocytes

Next, we analyzed the effects of irisin on ATP levels in LPS-stimulated cardiomyocytes, and its relationship with Fundc1-related mitophagy. ATP levels were significantly reduced in LPS-stimulated cardiomyocytes compared to the control group, but these effects were reversed by irisin (Figure 2(a)). Next, we analyzed the relationship between Fundc1-related mitophagy and irisin-mediated upregulation of ATP levels in LPS-stimulated cardiomyocytes by transfecting H9C2 cells with siRNA against Fundc1. Then, we analyzed ATP levels in the presence and absence of Fundc1. As shown in Figure 2(a), the ATP levels were significantly reduced in irisin-treated Fundc1-silenced cardiomyocytes compared to the irisin-treated cardiomyocytes alone. These results demonstrated that irisin enhanced ATP production in LPS-stimulated cardiomyocytes via Fundc1-related mitophagy.

RETRACTED

We then analyzed the activities of mitochondrial respiration complexes that regulate mitochondrial ATP production. LPS treatment significantly reduced the activity of mitochondrial respiration complexes I and III compared to the control group, but these effects were reversed by irisin (Figures 2(b) and 2(c)). However, the beneficial effects of irisin on the activities of complex I/III were abolished by Fundc1 silencing (Figures 2(b) and 2(c)). Decreased mitochondrial ATP production is closely associated with increased production of lactic acid, a by-product of glucose metabolism [50, 51]. Therefore, we analyzed changes in glucose and lactic acid levels in the medium of different experimental groups of cardiomyocytes. The levels of glucose were significantly higher, and lactic acid levels were significantly reduced in the growth medium of LPS-stimulated cardiomyocytes compared to the control group (Figures 2(d) and 2(e)). This suggested an arrest in mitochondrial oxidative phosphorylation. However, irisin treatment increased the levels of lactic acid and decreased glucose levels in the medium of LPS-stimulated cardiomyocytes (Figures 2(d) and 2(e)). This demonstrated that irisin promoted glucose metabolism in the LPS-stimulated cardiomyocytes. However, the beneficial effects of irisin on glucose metabolism were abolished by Fundc1 knockdown. Overall, these results demonstrated that irisin enhanced mitochondrial metabolism and ATP production in LPS-stimulated cardiomyocytes through Fundc1-related mitophagy.

### 3.3. Oxidative Stress Is Attenuated by Irisin through Fundc1-Related Mitophagy

Impaired mitochondrial metabolism is closely associated with mitochondrial oxidative stress [52–54]. Therefore, we analyzed the effects of irisin on oxidative stress in LPS-stimulated cardiomyocytes and the role of Fundc1-related mitophagy. The levels of ROS were significantly increased in the LPS-stimulated cardiomyocytes compared to the control group (Figures 3(a) and 3(b)). Irisin treatment suppressed the levels of ROS in LPS-stimulated cardiomyocytes, but these effects were abrogated by Fundc1 knockdown (Figures 3(a) and 3(b)). In addition to ROS production, we also measured the levels of antioxidative enzymes, such as GSH, SOD, and GPX in the cardiomyocytes. The activities of GSH, SOD, and GPX were significantly reduced in the LPS-stimulated cardiomyocytes compared to the control group (Figures 3(c)–3(e)), thereby suggesting decreased antioxidative capacity. Irisin treatment increased the activities of GSH, SOD, and GPX in LPS-stimulated cardiomyocytes, but these effects were abolished by Fundc1 silencing (Figures 3(c)–3(e)). These data suggested that the antioxidative capacity of LPS-stimulated cardiomyocytes was enhanced by irisin through a mechanism related to Fundc1-related mitophagy. Taken together, our results demonstrated that irisin suppressed oxidative stress in LPS-stimulated cardiomyocytes via Fundc1-related mitophagy.

RETRACTED

### 3.4. Mitochondria-Mediated Cardiomyocyte Death Is Inhibited by Irisin through Fundc1-Related Mitophagy

Mitochondrial ATP reduction and oxidative stress promote cardiomyocyte apoptosis by activating the mitochondria-dependent programmed cell death pathway [55–57]. Therefore, we analyzed if irisin attenuated cardiomyocyte apoptosis by activating Fundc1-related mitophagy. We used TUNEL staining assay to analyze the number of apoptotic cardiomyocytes in response to irisin treatment under LPS stress. The percentage of TUNEL-positive cardiomyocytes (apoptotic cells) was significantly higher in the LPS-stimulated group compared to the control group (40% vs. 10%; Figures 4(a) and 4(b)). Irisin significantly reduced the number of TUNEL-positive LPS-stimulated cardiomyocytes, but these effects were reversed by Fundc1 silencing (15% vs. 45%; Figures 4(a) and 4(b)). Taken together, these results suggested that LPS-stimulated cardiomyocyte apoptosis was inhibited by irisin through activation of Fundc1-related mitophagy. We then analyzed caspase-9 activity in LPS-stimulated cardiomyocytes. The activity of caspase-9 was significantly higher in LPS-stimulated H9C2 cells compared to the control group, but was significantly reduced by irisin treatment (Figure 4(c)). However, silencing of Fundc1 abolished the effects of irisin on caspase-9 (Figure 4(c)). Furthermore, caspase-3 activity was significantly elevated in LPS-stimulated cardiomyocytes but was reduced by irisin treatment in Fundc1-dependent manner (Figure 4(d)). However, knockout of Fundc1 increased caspase-3 activation in irisin-treated LPS-stimulated H9C2 cardiomyocytes (Figure 4(d)). These data confirmed that mitochondria-dependent apoptosis was inhibited by irisin in LPS-stimulated cardiomyocytes via Fundc1-dependent mitophagy.

RETRACTED

## 4. Discussion

Cardiac dysfunction is associated with increased morbidity and mortality in sepsis patients. Sepsis is a systemic inflammatory response that significantly reduces cardiac output and contributes to septic cardiomyopathy [58]. The risk factors associated with septic cardiomyopathy include upregulation of cytokines, hemodynamics disorder, sympathetic activation, decreased urine output, rapid rise in body temperature, and a sharp decrease in blood pressure [59]. However, therapeutic drugs are not available for the treatment of septic cardiomyopathy because molecular mechanisms underlying sepsis-related myocardial dysfunction are not well known [60]. Our previous studies suggested that mitochondrial fission was a potential mechanism that triggered cardiomyocyte apoptosis during LPS-induced sepsis. Therefore, mitochondrial damage was probably a key feature of septic cardiomyopathy. In this study, we demonstrated that Fundc1-related mitophagy was suppressed in LPS-stimulated cardiomyocytes. We also demonstrated that irisin administration restored mitophagy and attenuated mitochondrial dysfunction by increasing mitochondrial ATP production, suppressing mitochondrial oxidative stress, and inhibiting mitochondria-dependent pathway of cardiomyocyte apoptosis. This suggested that sepsis-related myocardial dysfunction may be effectively treated by targeting mitochondrial homeostasis.

Mitophagy promotes degradation of damaged mitochondrial components and is critical for maintaining mitochondrial homeostasis [61–63]. Mitophagy activation prevents ischemia-reperfusion injury by modulating oxidative stress and inflammation response [63]. Mitophagy activation also reduces calcium deposition from the vascular smooth muscle cells via AMPK/Opa1 signaling pathway [64]. Besides, hypoxia-related hypertension is attenuated by mitophagy through endothelial uncoupling protein 2 [65]. High-fat-diet impairs cardiac contraction by inactivating mitophagy [66]. Mitophagy activation improves endothelial dysfunction and microvascular damage by activating antioxidative, anti-inflammatory, and antiapoptotic mechanisms [18, 67]. In the present study, mitophagy induction through irisin treatment increased ATP content and attenuated oxidative stress and apoptosis in the LPS-stimulated cardiomyocytes. This suggested that induction of mitophagy was a potential mechanism to improve cardiomyocyte function in patients with sepsis.

RETRACTED

In the present study, we used irisin to improve cardiomyocyte function and survival by modulating mitophagy. The cardioprotective actions of irisin have also been previously reported. For example, serum irisin levels were reduced in diabetic patients and negatively correlated with cardiovascular events [68]. In type 2 diabetes model mice and hepatocytes, irisin inhibited hepatic gluconeogenesis and increased glycogen synthesis through the PI3K/Akt pathway [69]. Yin et al. reported that irisin acted as a mediator between obesity and vascular inflammation [70]. Furthermore, supplementation of irisin delayed progression of carotid atherosclerosis in dialysis patients [71]. Moreover, irisin improved endothelial proliferation through miRNA126-5p. In the present study, we demonstrated that irisin restored Fundc1-related mitophagy in LPS-stimulated cardiomyocytes as a model of sepsis cardiomyopathy.

There are several limitations in the present study. Our findings were not confirmed in animal models. Moreover, we did not investigate the association between mitophagy and inhibition of mitochondrial fission. Therefore, future investigations are required to confirm our findings and establish clinical relevance of irisin for treatment of septic cardiomyopathy.

In conclusion, our study demonstrates that irisin improved mitochondrial function and survival of LPS-stimulated cardiomyocytes via Fundc1-related mitophagy.

## Figures and Tables

**Figure 1:** Irisin activates Fundc1-related mitophagy in LPS-stimulated cardiomyocytes. (a, b) Western blot analysis shows Fundc1 levels in control, LPS-stimulated, and irisin plus LPS-stimulated cardiomyocytes. (c, d) Immunofluorescence assay results demonstrate mitophagy index in control, LPS-stimulated, and irisin plus LPS-stimulated cardiomyocytes. Note: ^∗^ denotes *p* < 0.05 vs. PBS group; ^#^ denotes *p* < 0.05 vs. LPS group; bar: 45 *μ*m.

**Figure 2:** Irisin enhances mitochondrial metabolism and ATP production in LPS-stimulated cardiomyocytes through Fundc1-related mitophagy. (a) ELISA analysis shows ATP levels in control, LPS-stimulated, irisin plus LPS-stimulated cardiomyocytes, and irisin plus LPS-stimulated Fundc1-silenced cardiomyocytes. (b, c) ELISA results show activities of mitochondrial complexes I and III in control, LPS-stimulated, irisin plus LPS-stimulated cardiomyocytes, and irisin plus LPS-stimulated Fundc1-silenced cardiomyocytes. (d, e) ELISA results show the levels of (d) glucose and (e) lactic acid in the medium from control, LPS-stimulated, irisin plus LPS-stimulated H9C2 cardiomyocytes, and irisin plus LPS-stimulated Fundc1-silenced cardiomyocytes. ^∗^ denotes *p* < 0.05 vs. PBS group; ^#^ denotes *p* < 0.05 vs. LPS group; ^@^ denotes *p* < 0.05 vs. LPS + irisin.

RETRACTED

**Figure 3:** Irisin attenuates oxidative stress in LPS-stimulated cardiomyocytes through Fundc1-related mitophagy. (a, b) Immunofluorescence assay results show ROS levels in control, LPS-stimulated, irisin plus LPS-stimulated cardiomyocytes, and irisin plus LPS-stimulated Fundc1-silenced cardiomyocytes. (c–e) ELISA assay results show activities of antioxidant enzymes, GSH, SOD, and GPX in the control, LPS-stimulated, irisin plus LPS-stimulated cardiomyocytes, and irisin plus LPS-stimulated Fundc1-silenced cardiomyocytes. ^∗^ denotes *p* < 0.05 vs. PBS group; ^#^ denotes *p* < 0.05 vs. LPS group; ^@^ denotes *p* < 0.05 vs. LPS + irisin; bar: 85 *μ*m.

**Figure 4:** Mitochondria-mediated cardiomyocyte death is inhibited by irisin through Fundc1-related mitophagy. (a, b) TUNEL assay results show the percentages of apoptotic cells in control, LPS-stimulated, irisin plus LPS-stimulated cardiomyocytes, and irisin plus LPS-stimulated Fundc1-silenced cardiomyocytes. (c, d) ELISA assay results show caspase-9 and caspase-3 activities in control, LPS-stimulated, irisin plus LPS-stimulated cardiomyocytes, and irisin plus LPS-stimulated Fundc1-silenced cardiomyocytes. ^∗^ denotes *p* < 0.05 vs. PBS group; ^#^ denotes *p* < 0.05 vs. LPS group; ^@^ denotes *p* < 0.05 vs. LPS + irisin group; bar: 120 *μ*m.

## Data Availability

The analyzed data sets generated during the present study are available from the corresponding author on reasonable request.
